# Identification of Novel Biomarkers Related to Lung Squamous Cell Carcinoma Using Integrated Bioinformatics Analysis

This article has been retracted.

**DOI:** 10.1155/2021/9059116

**Published:** 2021-10-08

**Authors:** Haiyan Wang, Lizhi Huang, Li Chen, Jing Ji, Yuanyuan Zheng, Zhen Wang

**Affiliations:** ^1^Department of Ultrasonography Center, Tai'an City Central Hospital, Tai'an, China; ^2^Department of Thoracic Surgery, Shenzhen Bao'an People's Hospital (Group), Shenzhen, China; ^3^Department of Vascular, Tai'an City Central Hospital, Tai'an, China; ^4^Department of Geriatrics, Tai'an City Central Hospital, Tai'an, China; ^5^Department of Radiotherapy, Tai'an City Central Hospital, Tai'an, China; ^6^Department of Thoracic Oncology, Sun Yat-sen University Cancer Center, Guangzhou, China

## Abstract

**Background:**

Lung squamous cell carcinoma (LUSC) is one of the most common types of lung carcinoma and has specific clinicopathologic characteristics. In this study, we screened novel molecular biomarkers relevant to the prognosis of LUSC to explore new diagnostic and treatment approaches for this disease.

**Methods:**

We downloaded GSE73402 from the Gene Expression Omnibus (GEO) database. GSE73402 contains 62 samples, which could be classified as four subtypes according to their pathology and stages. Via weighted gene coexpression network analysis (WGCNA), the main module was identified and was further analyzed using differentially expressed genes (DEGs) analysis. Then, by protein-protein interaction (PPI) network and Gene Expression Profiling Interactive Analysis (GEPIA), hub genes were screened for potential biomarkers of LUSC.

**Results:**

Via WGCNA, the yellow module containing 349 genes was identified, and it is strongly related to the subtype of CIS (carcinoma in situ). DEGs analysis detected 180 genes that expressed differentially between the subtype of CIS and subtype of early-stage carcinoma (Stage I and Stage II). A PPI network of DEGs was constructed, and the top 20 genes with the highest correlations were selected for GEPIA database to explore their effect on LUSC survival prognosis. Finally, ITGA5, TUBB3, SCNN1B, and SERPINE1 were screened as hub genes in LUSC.

**Conclusions:**

ITGA5, TUBB3, SCNN1B, and SERPINE1 may have great diagnostic and prognostic significance for LUSC and have great potential to be new treatment targets for LUSC.

## 1. Introduction

Lung cancer is the most common cause of cancer-related deaths around the world; its morbidity also ranks first around all cancer types. Lung squamous cell carcinoma (LUSC) is a common type of lung cancer, which has specific clinicopathologic characteristics compared with the other types due to differences in their origin of cells [1, 2]. The pathogenesis of LUSC is complicated and is involved in large numbers of molecular and cellular events, but unfortunately, the majority of these events still remain to be explored [3, 4]. These reasons cause unsatisfactory treatment outcomes in LUSC, leading to the median survival approximately 30% inferior to the other lung cancer types [1, 5, 6].

Surgery and chemoradiotherapy remain the main treatment of lung cancer in the past several decades, while with the development of genomics, large amounts of molecular biomarkers participating in the tumorigenesis, progression, metastasis, and drug resistance have been detected [7]. EGFR-TKI (epidermal growth factor receptor-tyrosine kinase inhibitor) and ALK (anaplastic lymphoma kinase) inhibitors are the best of these developments and have changed clinical treatment mode of lung cancer, especially in the treatment of lung adenocarcinoma (LUAD) [4, 8–11]. Unfortunately, these targets are not successful in LUSC, because the abovementioned mutations/alterations are rare in LUSC [6, 10–12].

Therefore, molecular mechanism-related researches will play key roles in prediction and treatment of LUSC, and a great portion of them have been reported recently. Mascaux et al. reported that pulmonary tumorigenesis involves a series of coactions of preinvasive bronchial epithelial cells and immunocytes, which indicated that immune biomarkers for early diagnosis and immunotherapy for individuals at high risk awaited to be uncovered [13]. Momcilovic et al. discovered that adaptive glutamine metabolism was regulated by GSK3 signaling axis in LUSC, which may be a prediction for response to combined metabolic therapies targeting mTOR and glutaminase [14]. Huang et al. reported that YAP could inhibit disease progression by deregulation of the DNp63-GPX2 axis and ROS accumulation in LUSC, which may be a potential to improve precision medicine of patient with LUSC [15]. Furthermore, with the development of bioinformatics in recent years, it is accessible for us to explore the whole molecular alterations in tumors at multiple levels including DNA, epigenetic modification, RNA, and proteins [16]. Via weighted gene coexpression network analysis (WGCNA), Niemira et al. found that CCNB2 and GNG11 are novel biomarkers contained in modules connected with tumor size, PET/CT SUVmax, and recurrence-free survival (RFS) in LUSC [17]. By analyzing datasets online, Gao et al. detected a couple of biomarkers related to development and prognosis of LUSC, including FEN1, CCNA2, AURKA, and AURKB [18]. Although lots of studies have reported some biomarkers that may be involved in pathogenesis or progression of LUSC, more biomarkers are waiting to be discovered to construct a complete understanding of LUSC. Hence, in order to decrease LUSC-related deaths and optimize treatment mode of LUSC, the detection of more novel biomarkers in LUSC is still required.

In this study, we downloaded GSE73402 from the Gene Expression Omnibus (GEO) database, which is a public database for high-throughput microarray and next-generation sequence functional genomic data sets submitted by the research community worldwide. GSE73402 contains 62 samples, including precancerous progression cases and lung squamous carcinoma cases, which could display transcriptome profiles of all stages of lung squamous carcinoma. Firstly, we constructed coexpression modules using weighted gene coexpression network analysis (WGCNA) and found the main module. Secondly, via differentially expressed genes (DEGs) analysis, protein-protein interaction (PPI) network, and Gene Expression Profiling Interactive Analysis (GEPIA), hub genes were screened for potential biomarkers of LUSC. In this study, we applied WGCNA to construct coexpression network for exploring tumorigenesis and development of lung squamous carcinoma for the first time and identified the main module and hub genes. The workflow of our study is shown in Figure 1.

## 2. Materials and Methods

### 2.1. Data Information

The gene expression profile of GSE73402 was searched in NCBI GEO website with “Lung squamous cancer” and “Homo sapiens” as keywords. GSE73402 consists of 80 cases, including 23 precancerous cases [5 cases with mild or moderate dysplasia (P1) and 18 cases with carcinoma in situ (P2)] and 39 lung squamous carcinoma cases (11 Stage I, 13 Stage II, 8 Stage III, and 7 Stage IV cases), and the platform of this series is GPL17077 (Agilent-039494 SurePrint G3 Human GE v2 8x60K Microarray 039381) [19]. According to pathology and stages of these samples, we classified them as 4 subtypes, which are dysplasia (mild or moderate dysplasia), CIS (carcinoma in situ), early-stage carcinoma (Stage I and Stage II), and advanced carcinoma (Stage III and Stage IV).

### 2.2. Construction of WGCNA

In this section, top 5,000 genes were selected according to average expression and then were calculated by WGCNA algorithm [20]. First, the scale-free topology fit index for powers was calculated and the soft threshold for network construction was selected. Then, the scale-free network was constructed and the module eigengene (ME) of each module was calculated. Finally, the correlation between ME and pathological trait of each module was calculated, and gene significance (GS) of genes in the main module was further calculated [21].

### 2.3. Gene Ontology (GO) and Pathway Enrichment Analysis

To explore biological functions of genes contained in the main module, Gene Ontology (GO), Disease Ontology (DO), and Kyoto Encyclopedia of Genes and Genomes (KEGG) pathway enrichment analysis were performed based on the package GDCRNATools of R/Bioconductor software [22–25]. *p* value < 0.05 was considered statistically significant.

### 2.4. Differentially Expressed Genes (DEGs) Analysis

In the previous section, correlation coefficient between yellow module and carcinoma in situ (CIS) ranked first. CIS is an intermediate status between dysplasia and invasive carcinoma, and it has great potential to progress to invasive disease [26]. So by virtue of DEGs analysis between CIS and early-stage carcinoma specimens, we could further screen genes in yellow module. DEGs were analyzed using limma package of R/Bioconductor software with adjusted *p* value < 0.05 and ∣logFC | >1 [27]. Then, top 25 upregulated and top 25 downregulated DEGs were selected to draw heat maps.

### 2.5. Protein-Protein Interaction Network Analysis

DEGs were then mapped to NetworkAnalyst database, which could provide a visual network to help understand complex molecular interactions and has a function of human tissue-specific PPI analysis [28]. So, we mapped DEGs using Cytoscape software and screened the top 20 genes with the most relevance [29].

### 2.6. Survival and mRNA Expression Analysis

In this section, we made use of boxplot to visualize the mRNA expression of hub genes between LUSC tissues and normal lung tissues by utilizing Gene Expression Profiling Interactive Analysis (GEPIA) database, which was a website aiming at analyzing gene expression data from GTEx (Genotype-Tissue Expression) and TCGA (The Cancer Genome Atlas) projects [30]. Furthermore, we kept using GEPIA database to assess the association between expression levels of hub genes and prognosis. Finally, biomarkers associated with mRNA expression differences or survival differences were selected.

### 2.7. Drugs Targeting Hub Genes and Genetical Alterations of Hub Genes

Approved drugs targeting hub genes directly were explored utilizing NetworkAnalyst database, which collected information from the DrugBank database (Version 5.0) [28, 31]. We further explored genetic alterations of hub genes via cBio Cancer Genomics Portal (cBioPortal), which could provide a bulk of cancer genomic datasets of various cancers and enabled us to compare genetic alterations across different samples [32].

## 3. Results

### 3.1. Preprocessing of Microarray Data

The data of GSE73402 was searched and downloaded from GEO database and then was processed by R packages. We annotated probes in series matrix files by using gene symbol information from soft formatted family files. In this section, gene symbols and probes were matched, the probe annotated by more than one gene was deleted, and the average value was calculated and recorded as the final expression value for the gene matched by multiple probes. Finally, 31,998 genes were matched and retained in expression matrix [33].

### 3.2. Construction of Weighted Coexpression Network

Standard deviation (SD) of each gene was calculated and ranked in decreasing order; top 5,000 genes were selected for WGCNA. Then, the optimal power value was selected, which would affect scale independence and mean connectivity of gene coexpression module. As we see in Figure 2(a), when the power value was 3, a relatively balanced scale independence and mean connectivity could be gotten. Coexpression module was analyzed using the top 5,000 genes and selected top 5,000 genes, and 13 gene coexpression modules were constructed finally (Figure 2(b)). All modules were marked with different colors and ranked according to gene numbers (Figure 2(c)) [7, 33].

### 3.3. Detection and Function Enrichment Analysis of Key Module

According to pathology and stages of samples from GSE73402, we classified these samples as 4 subtypes, which are dysplasia (mild or moderate dysplasia), CIS (carcinoma in situ), early-stage carcinoma (Stage I and Stage II), and advanced carcinoma (Stage III and Stage IV). Through module-feature relationship analysis, we identified that CIS was strongly associated with the yellow module (*r* = 0.6, *p* = 3*E* − 7) (Figure 3(a)) [20, 34]. Scatter plot of gene significance versus module membership for yellow module is shown in Figure 3(b). Considering that CIS is an intermediate status between dysplasia and invasive carcinoma, genes contained in yellow module may play vital roles in tumorigenesis and progression of LUSC [26].

Therefore, we focused on the function and pathway of genes contained in yellow module next. Because the yellow module contained both mRNA, lncRNA, and the RNAs without official symbol, so we transformed gene names from gene symbol to gene stable ID using BioMart database [35]. Yellow module contained 349 genes; 284 of them were transformed to gene stable ID for enrichment analysis. Function and pathway enrichment analysis of these genes was conducted by GDCRNATools, an R/Bioconductor package [22]. Top 25 Gene Ontology (GO), Disease Ontology (DO), and Kyoto Encyclopedia of Genes and Genomes (KEGG) pathway enrichment analysis were showed in bubble diagram (Figure 4). As we see in the figure, biological process (BP) of GO shows that genes are gathered in “hormone metabolic process”, “cellular hormone metabolic process”, “neural precursor cell proliferation”, and “positive regulation of synaptic transmission”. For molecular function (MF), the genes are gathered in “hormone binding” and “sulfotransferase activity”. For cellular component (CC), the genes are gathered in “presynapse”, “apical part of cell”, “apical plasma membrane”, “axon part”, and “receptor complex”. KEGG pathway enrichment analysis shows that the genes are enriched in “glycolysis/gluconeogenesis”, “fatty acid degradation”, “tyrosine metabolism”, and “tryptophan metabolism”. DO enrichment analysis indicated that the genes are mainly related to “endocrine gland cancer” and “lung carcinoma”.

### 3.4. Identification of DEGs between CIS and Early-Stage Carcinoma

GSE73402 contains 62 cases, of which 18 cases are carcinoma in situ (CIS) and 24 cases are early-stage carcinoma (11 Stage I, 13 Stage II). Genes in yellow module were further screened using limma package in R, and adjusted *p* value < 0.05 and ∣log2FC | >1 were considered as statistical significance. 180 genes expressing differentially were detected, including 67 upregulated genes and 113 downregulated genes. The top 25 upregulated genes and downregulated genes were chosen for next analysis and shown in heat map (Figure 5).

### 3.5. PPI Network Construction

All DEGs were submitted into the NetworkAnalyst database using lung tissue-specific analysis. The most significant subnetwork contains 58 genes of all DEGs submitted (seeds), 932 nodes, and 1,067 edges. The PPI network of the most important subnetwork is shown in Figure 6. The top 20 genes with the highest correlations are shown in Table 1 and are chosen for the next analysis.

### 3.6. Detection of Hub Genes by GEPIA

The mRNA expression level and survival data of hub genes selected above was further analyzed using GEPIA website. Results indicated that 6 genes expressed differently in lung squamous cell cancer compared with normal lung samples (*p* < 0.05), which were CA9, CCT3, ITGA5, TUBB3, ADRB2, and SCNN1B (Figure 7(a)). Survival analysis indicated that high expression level of TUBB3 and ITGA5 was remarkably associated with worse overall survival for patients with LUSC (*p* < 0.05, Figure 7(b)), and high expression level of SCNN1B was approximately associated with worse overall survival for these patients (*p* = 0.091, Figure 7(b)). While the expression level of CA9, CCT3, and ADRB2 had no statistical significance with overall survival of these patients. It is interesting that mRNA expression of SERPINE1 did not show difference between tumor and normal tissues, but its mRNA expression level in tumors was associated with overall survival in patients with LUSC (*p* < 0.05, Figure 7(b)). Therefore, ITGA5, TUBB3, SCNN1B, and SERPINE1 can be regarded as hub genes with great diagnostic and prognostic significance for LUSC.

### 3.7. Drugs Targeting Hub Genes and Genetical Alterations of Hub Genes

Via protein-drug interactions in NetworkAnalyst, 15 drugs targeting the hub genes directly were searched, of which 8 drugs for SERPINE1, 5 drugs for TUBB3, and 2 drugs for SCNN1B (Table 2), while there is no drug that can target ITGA5 directly as far as we know. OncoPrint of cBioPortal is shown in Figure 8(a), which indicates alteration statuses of 4 hub genes in TCGA patients with LUSC. All 4 genes altered in 86 (7%) of all 1176 patients, and SERPINE1 altered most (5%) compared with the other genes. Amplification and missense mutation are the main alteration type, and the detailed alteration type of all 4 genes is shown in Figure 8(b).

## 4. Discussion

Although a mass of studies have made efforts in diagnosis and treatment of lung cancer, LUSC still lacks effective therapeutic target and prognostic predictor, resulting in poor survival of patients with LUSC [1]. In order to improve diagnosis and treatment of LUSC, it is necessary to keep exploring molecular mechanisms related to tumorigenesis and progression in LUSC. Thankfully, with the development of bioinformatics recently, it is accessible for us to explore the whole molecular events in tumors at multiple levels involving DNA, epigenetic modification, RNA, and proteins, which could indicate novel biomarkers for diagnosis, treatment, and prognosis prediction of specific tumors [16, 36].

To detect new biomarkers that have clinical significance in LUSC, we searched and applied one profile dataset from GEO website: GSE73402. GSE73402 consists of 80 cases, including 23 precancerous cases [5 cases with mild or moderate dysplasia (P1) and 18 cases with carcinoma in situ (P2)] and 39 lung squamous carcinoma cases (11 Stage I, 13 Stage II, 8 Stage III, and 7 Stage IV cases), which represents the whole process of tumorigenesis and development in LUSC. Hence, via analyses of WGCNA, we detected that a gene list (yellow module) was strongly associated with the subtype of carcinoma in situ (CIS). Considering carcinoma in situ plays a vital role in the process of carcinoma, genes contained in yellow module may be further screened as novel biomarkers for diagnosis and treatment in LUSC. Then, in a series of analyses via enrichment analysis, DEGs, PPI, GEPIA, and cBioPortal, 4 genes (ITGA5, TUBB3, SCNN1B, and SERPINE1) were detected as biomarkers associated with the prognosis of LUSC.

In our study, TUBB3 was found to be associated with survival in LUSC, and its high expression predicted worse survival. TUBB3 gene of Homo sapiens is located on chromosome 16q24.3 and is composed of 4 exons. It encodes a protein of 450aa, beta-III tubulin, which is the main component of microtubules and has a GTPase domain that is necessary for regulating microtubule dynamics [37]. Due to the vital function of microtubules in tumorigenesis and progression of carcinoma, many studies have focused on this gene and its effect on cancer treatment [37]. Kamath et al. reported that overexpression of beta-III tubulin could reduce the ability of paclitaxel to suppress microtubule dynamics and thus induce paclitaxel resistance, which could result in a poor survival prognosis for patients [38]. Levallet et al. found that the expression of TUBB3 was an independent prognostic factor for patients with early non-small-cell lung cancer who were treated by preoperative chemotherapy, and K-Ras mutations were determinants in regulating TUBB3 expression [39].

Human SCNN1B gene is located on chromosome 16p12.2 and its encoding production is *β*-subunit of the epithelial sodium channel (ENaC), which is a multiprotein complex composed of three subunits (*α*, *β*, and *γ*) and is in charge of fluid and electrolyte transport across epithelia. Although SCNN1B is regarded as a membrane channel in the past, a series of studies have indicated that SCNN1B also involves in cellular differentiation [40, 41]. Qian et al. reported that SCNN1B expression could be silenced commonly via promoter hypermethylation in gastric cancer (GC) cell lines and primary tumor tissues, and indicated that GRP78 overexpression could eliminate the inhibitory effect of SCNN1B on cell growth and migration and thus promoted tumor progress [41]. Dalgin et al. detected hypermethylation of SCNN1B in renal cell carcinoma and suggested that it may serve as a feasible diagnostic test of urine and blood samples [42]. In our study, SCNN1B mRNA expression level in tumor tissues is lower than that in normal lung tissues, which is consistent with previous studies and indicates that SCNN1B may be hypermethylated in LUSC. All studies mentioned above showed that SCNN1B may act as a tumor suppressor, but in GEPIA database, the patients with high SCNN1B mRNA expression level suffer a poor survival prognosis (*p* = 0.091). Therefore, more studies are required to explore the molecular mechanism of SCNN1B in LUSC and to confirm its role playing in LUSC survival prognosis.

Human gene SERPINE1 (serpin family E member 1) is located on chromosome 7q22.1, and it encodes plasminogen activator inhibitor-1 (PAI-1), which is an inhibitor of tissue plasminogen activator (tPA) and urokinase (uPA), and involves in fibrinolysis [43].

The plasminogen activator system can affect cell migration and angiogenesis, so it not only controls the intravascular fibrin deposition but also participates in a series of biological processes, including tumor growth, invasion, and metastasis [44]. Wang et al. found that via interacting with LRP1, overexpression of PAI-1 might enhance invasion and migration of ESCC cells [45]. Xu et al. detected that PAI-1 expression significantly increased in breast tumor tissues compared with the normal tissues, and the expression level was relevant to prognosis of patients with triple negative breast cancer [46]. Lin et al. reported that PAI-1 could promote epithelial-mesenchymal transition (EMT) in NSCLC cells by activating the STAT3 signaling pathway, which indicated that PAI-1 could be a biomarker for prognosis prediction and a potential therapeutic target [47]. Analysis of GSE73402 in our study also shows that SERPINE1 mRNA expression is elevated in invasive lung squamous carcinoma compared with carcinoma in situ. And the patients with high level of SERPINE1 mRNA expression suffer a poor survival via GEPIA database, which is consistent with previous studies.

ITGA5 gene of Homo sapiens is located on chromosome 12q13.13 and encodes integrin alpha 5, which is a member of integrin alpha chain family. Integrins are heterodimeric integral membrane proteins and consist of an alpha subunit and a beta subunit that enable integrins to function in cell signaling and surface adhesion [43]. Integrins have been reported that it may involve in angiogenesis and lymphangiogenesis and may be a potential therapeutic target for inhibition of tumor angiogenesis, lymphangiogenesis, and metastasis [48]. Yu et al. indicated that ITGA5 overexpression could accelerate the progression of colorectal cancer (CRC) and that was closely associated with its enhanced O-GlcNAcylation [49]. Feng et al. found that ITGA5 might work as a facilitator in glioblastoma (GBM), and miR-330-5p could inhibit proliferation and invasion of GBM cells through targeting ITGA5 [50]. Xiao et al. reported that miR-205 reexpression could downregulate ITGA5 expression and thus impaired TNBC cell metastatic traits, which suggested that miR-205 and ITGA5 may be potential biomarkers for treatment of metastatic TNBC [51]. Our analysis shows that ITGA5 mRNA expression increases in invasive lung squamous carcinoma compared with carcinoma in situ; despite it is contrary to the outcome from GEPIA database, ITGA5 is still identified as a risk factor for survival of patients with LUSC in our study.

## 5. Conclusion

In conclusion, we utilized a series of comprehensive bioinformatics analyses including weighted gene coexpression network analysis (WGCNA), differentially expressed genes (DEGs), and subsequent online analyses. Finally, ITGA5, TUBB3, SCNN1B, and SERPINE1 are screened as hub genes with great diagnostic and prognostic significance for LUSC and have great potential to be new treatment targets for LUSC. In consideration of the fact that all analyses and results in our study are based on bioinformatics database and methodology, the mechanism of these genes on tumorigenesis and progression of LUSC remains to be elucidated.

## Figures and Tables

**Figure 1:** Workflow of this study. WGCNA: weighted gene coexpression network analysis; DEGs: differentially expressed genes; PPI: protein-protein interaction network.

**Figure 2:** Gene coexpression module construction. (a) Scale-free fit index and the mean connectivity for soft thresholding powers. (b) Gene dendrogram and module colors. (c) Number of genes in each gene coexpression module.

**Figure 3:** Module-feature relationships. (a) Heat map of correlations between sample subtypes and MEs (corresponding Pearson correlation and *p* value). (b) The module membership (MM) versus gene significance (GS) scatter plot for CIS in yellow module. MEs: module eigengenes; CIS: carcinoma in situ.

**Figure 4:** Functional and pathway enrichment analysis of genes in yellow module. (a) GO-BP enrichment analysis. (b) GO-MF enrichment analysis. (c) DO enrichment analysis. (d) KEGG pathway enrichment analysis. GO: Gene Ontology; BP: biological process; MF: molecular function; DO: Disease Ontology; KEGG: Kyoto Encyclopedia of Genes and Genomes.

**Figure 5:** Expression heat map of DEGs between carcinoma in situ (CIS) and early-stage carcinoma (Stage I and Stage II). (a) Expression heat map of top 25 upregulated genes. (b) Expression heat map of top 25 downregulated genes. DEGs: differentially expressed genes.

**Figure 6:** DEGs are mapped using lung tissue-specific PPI analysis in NetworkAnalyst database. The red-filled hexagon node represents for the 20 proteins with the largest number of effector proteins.

**Figure 7:** (a) Six genes expressed differently in LUSC compared with normal lung samples using GEPIA database (^∗^*p* < 0.05). (b) Expression level of 4 genes is associated with overall survival for patients with LUSC using GEPIA database. LUSC: lung squamous cell cancer; GEPIA: Gene Expression Profiling Interactive Analysis.

**Figure 8:** (a) A visual summary showing genetic alterations of 4 hub genes in TCGA patients with LUSC. (b) Specific alteration types of 4 hub genes. TCGA: The Cancer Genome Atlas Program.

**Table 1:** The top 20 DEGs with the largest number of effector proteins.

Label	Degree	Betweenness
ADRB2	233	257445.1
PTN	106	92928.5
CCT3	77	81739.98
TUBB3	59	62695.01
TCEA2	54	47992.46
BAG2	50	44353.53
ATP4A	46	58624.97
ENO2	34	30455.94
ITGA5	27	22662.45
GHR	24	21186.87
CA9	23	24244.3
SDCBP2	20	17499
KRT4	20	14502.74
VAV3	18	13556.04
TRIM46	18	13101.6
SCNN1B	18	12939.94
EPHA4	15	11448.19
KRT24	15	10896.56
SERPINE1	15	10494.79
GLUL	14	10191.6

**Table 2:** The approved drugs targeting hub genes directly.

Gene ID	Approved drugs targeting the gene directly
SCNN1B	Amiloride
	Triamterene
TUBB3	ZEN-012
	CYT997
	Epothilone D
	Ixabepilone
	Epothilone B
SERPINE1	Alteplase
	Urokinase
	Reteplase
	Anistreplase
	Tenecteplase
	Drotrecogin alfa
	Troglitazone
	Plasmin

## Data Availability

The data used to support the findings of this study are available from the corresponding authors upon request.
